# Understanding the Cellular Sources of the Fractional Exhaled Nitric Oxide (FeNO) and Its Role as a Biomarker of Type 2 Inflammation in Asthma

**DOI:** 10.1155/2022/5753524

**Published:** 2022-05-02

**Authors:** Jose M. Escamilla-Gil, Mar Fernandez-Nieto, Nathalie Acevedo

**Affiliations:** ^1^Institute for Immunological Research, University of Cartagena, Cartagena 130014, Colombia; ^2^Servicio de Alergología Fundación Jiménez Díaz IIS CIBERES (Ciber de Enfermedades Respiratorias) Unidad Multidisciplinar de Asma, Madrid 28040, Spain

## Abstract

Fractional exhaled nitric oxide (FeNO) has gained great clinical importance as a biomarker of type 2 inflammation in chronic airway diseases such as asthma. FeNO originates primarily in the bronchial epithelium and is produced in large quantities by the enzyme inducible nitric oxide synthase (iNOS). It should be noted that nitric oxide (NO) produced at femtomolar to picomolar levels is fundamental for respiratory physiology. This basal production is induced in the bronchial epithelium by interferon gamma (IFN*γ*) via Janus kinases (JAK)/STAT-1 signaling. However, when there is an increase in the expression of type 2 inflammatory cytokines such as IL-4 and IL-13, the STAT-6 pathway is activated, leading to overexpression of iNOS and consequently to an overproduction of airway NO. Increased NO levels contributes to bronchial hyperreactivity and mucus hypersecretion, increases vascular permeability, reduces ciliary heartbeat, and promotes free radical production, airway inflammation, and tissue damage. In asthmatic patients, FeNO levels usually rise above 25 parts per billion (ppb) and its follow-up helps to define asthma phenotype and to monitor the effectiveness of corticosteroid treatment and adherence to treatment. FeNO is also very useful to identify those severe asthma patients that might benefit of personalized therapies with monoclonal antibodies. In this review, we revised the cellular and molecular mechanisms of NO production in the airway and its relevance as a biomarker of type 2 inflammation in asthma.

## 1. Introduction

The identification and use of biomarkers have acquired great importance in clinical practice, especially to identify phenotypes of chronic respiratory diseases such as asthma [1–4] Several studies demonstrate the cost-effectiveness of using these biomarkers compared to other clinical functional tests [5–8]. Fractional exhaled nitric oxide (FeNO) has been suggested as a noninvasive biomarker of airway inflammation [3, 9, 10]. FeNO can be measured in a standardized manner, with a constant expiratory flow breathing technique that determines nitric oxide (NO) levels in exhaled air [3]. Currently, FeNO can help to establish the diagnosis of asthma, predict response to inhaled steroids, and monitor the patient's response to inhaled steroids and the optimal dose for asthma control and also serves as an indicator of relevance for treatment with biological drugs [3, 4, 11–13]. FeNO is elevated in asthmatic patients with type 2 inflammation, as well as in other respiratory diseases such as allergic rhinitis and chronic rhinosinusitis with nasal polyposis [14–16]. In addition, FeNO increases with moisture, mold, and allergen exposure and is rapidly reduced with steroid treatment [17–22]. To properly interpret a FeNO measurement and its relevance in composite analysis with other type 2 biomarkers such as eosinophil cell counts or periostin, it is essential to understand the immune mechanisms of NO production in the airways. The aim of this study is to review the scientific literature about how exhaled NO is produced in the airways and its applications as biomarker of asthma.

## 2. Methodology

An integrative review of the scientific literature was performed by searching on the MEDLINE database using the PubMed search engine. Medical subject headings (MeSH) terms and synonyms were used as keywords in search strings: ((Fractional Exhaled Nitric Oxide) OR (FeNO) OR (FENO) OR (exhaled NO)) AND ((asthma) OR (type 2 inflammation) OR (biomarker)) ((Fractional Exhaled Nitric Oxide) OR (FeNO) OR (FENO) OR (exhaled NO)) AND ((cytokines) OR (iNOS) OR (synthesis)). No date restrictions were applied and included articles until February 2022. References found through manual search—including citations of the articles identified in the database search—were also taken in consideration. All retrieved articles were analyzed based on title, abstract, full-text content, and date of publication (for instance, if were first description or replication), and those related with the topic were included in this review.

## 3. Biochemistry and Synthesis of Nitric Oxide

NO is an odorless and colorless gas that is formed by the union of two oxygen (O_2_) and one nitrogen (N) atoms, being a small and neutral molecule with ability to diffuse freely through cell membranes [23]. Combining NO with superoxide produces other radicals, including peroxynitrite (ONOO^−^), nitrogen dioxide (NO_2_), and hydroxyls that injure cells. NO is synthesized from the amino acid L-arginine by nitric oxide synthase (NOS) enzymes, in a process dependent of oxygen and the coenzyme nicotinamide adenine dinucleotide phosphate (NADPH) [24]. NOS are expressed in 3 isoforms that were originally referred to as constitutive or inducible [23]. The constitutive isoforms are expressed in a wide variety of cells and are known as NOS1 (or neuronal, nNOS) and NOS3 (or endothelial, eNOS). The inducible form (iNOS), also known as NOS2, is expressed in several immune cells after stimulation by cytokines and proinflammatory signals, but it should be noted that under normal conditions iNOS is expressed at low levels in the epithelial cells of the human airway [25–27]. NOS use L-arginine as a substrate and molecular oxygen, and NADPH as cosubstrates, as well as flavin adenine dinucleotide (FAD), flavin mononucleotide (FMN), and (*6R*-) 5, 6, 7,8-tetrahydro-1-biopterin (BH4) as cofactors (Figure 1). NOS exists as homodimers with a terminal carboxyl reductase domain and an amino terminal oxygenase domain [28, 29]. When NOS monomers bind to calmodulin do occur an electron transference from the reductase domain to the oxygenase domain. The monomers of the constitutive NOS (nNOS and eNOS) require a high concentration of calcium to bind calmodulin, while iNOS binds with high affinity to calmodulin even in the absence of calcium [29]. This capacity of iNOS allows the production of NO at nanomolar levels, which are maintained for several hours and contribute to the pathophysiological effects of NO and its detectable elevation in exhaled air (Figure 2). When NO is produced in large quantities by iNOS, it reacts with superoxide anions (O2^−^) formed in the airway generating the formation of peroxynitrite (ONOO^−^), a powerful oxidizing agent that reacts with DNA, proteins, and cell membrane lipids, damaging and causing cell death. As we will mention later, elevated NO also affects the immune response by promoting type 2 inflammation [30].

iNOS is physiologically expressed in airway epithelial cells maintaining the baseline NO levels, in a process mediated by a homeostatic interferon gamma (INF*γ*) that is naturally produced in the fluid of the pulmonary epithelial lining and activates the Janus kinase signal pathway (JAK) and the signal transducer and transcription activator 1 (STAT-1). Activation of STAT-1 and subsequent induction of interferon-1 response factor (IRF-1) result in iNOS transcription and a constant synthesis of NO that is not affected by the action of corticosteroids **(**Figure 3**)** [31] . In healthy adults, baseline FeNO levels are between 10 and 17 parts per billion (ppb) with an average of 13 ppb [23, 32].

Elevated FeNO levels are detected in patients with acute or chronic airway inflammation including several asthma phenotypes [33]. This increase reflects the induction of iNOS by IL-4 and IL-13 in airway epithelial cells and inflammatory cells and is an indicator of alteration in the balance of cytokine signals. In respiratory infections of viral origin, an increase in FeNO is also observed, and although the mechanism is still unclear, it is believed that interferon-induced pathways activate the expression of iNOS in the epithelium of the airways [34]. Decreased FeNO levels have been observed in patients with cystic fibrosis, chronic obstructive pulmonary disease (COPD), neutrophilic asthma, bronchopulmonary dysplasia, and respiratory distress of the newborn (Figure 4) [33, 35].

The increased activity of iNOS favors the differentiation of Th2 lymphocytes and inhibits Th1 and Th17 with IL-4 and IL-13 perpetuating NO production and type 2 inflammation [36, 37]. NO inhibits IL-12 synthesis in activated macrophages, decreases aryl hydrocarbon receptor (AhR) expression, and is cytotoxic for memory Th1 lymphocytes [38–40]. NO also inhibits Th17 lymphocytes by nitration of tyrosine residues in the transcription factor ROR*γ*t and by reducing AhR expression [36, 41]. In contrast, low NO concentrations increase IL-12 receptor (IL-12R) expression, favoring the development of Th1 lymphocytes [42] and induce the development of Th17 cells [36, 42]. In fact, “knock-out” mice for iNOS have an increased Th1 response [37].

## 4. Cellular and Molecular Mechanisms of FeNO Elevation in Type 2 Inflammation

After the detection of NO in the exhaled air of humans, it was evidenced that atopic subjects had higher NO levels than nonatopic subjects. The main factor underlying this increase in NO is the high expression of iNOS by airway epithelial cells in atopic patients [34]. NO contributes to the inflammatory process via alterations in apoptosis, phagocytosis, and leukocyte adherence and increases the reactivity and recruitment of mast cells, basophils, lymphocytes, and eosinophils [30], thus promoting bronchial hyperreactivity and lung inflammation [30]. In fact, in murine models of asthma that are “knock-out” for all NOS isoforms show reduced eosinophilic infiltrates, reduced mucus hypersecretion, and lower concentrations of type 2 cytokines [43]. Treatment of asthmatic patients with corticosteroids increases or restores INF*γ* levels in bronchoalveolar lavage and bronchial epithelial cells and decreases FeNO levels [44, 45].

IL-4 induces iNOS expression in airway epithelial cells in the presence of INF*γ*, but when IL-4 expression occurs at abnormally high levels, signaling is skewed towards the JAK/STAT-6 pathway altering NO production [23, 46]. Altered expression of IL-13, a typical feature of type 2 inflammation, can also induce iNOS expression in the bronchial epithelium via STAT-6 pathway (Figure 5) [23, 32, 34, 47]. Modena et al. have found 549 genes whose expression in bronchial epithelial cells correlates with FeNO levels. High FeNO patients have a very characteristic pattern with overexpression of several genes involved type 2 inflammation pathways [48]. *NOS2* expression was the most correlated with FeNO levels (rho = 0.72, *P* value <10 ^−7^) which supports its effects on bronchial epithelium cells and the production of exhaled NO. Similarly, expression of type 2 inflammation genes such as periostin (*POSTN*), chlorine channel accessory 1 (*CLCA1*), and member 2 of the Serpin 2 family (*SERPINB2*) was also correlated with FeNO values (rho from 0.49 to 0.60, *P* < 10^−7^). In contrast, the mucin gene (*MUC5B*), which is strongly repressed by IL-13, has a negative correlation with FeNO levels [48]. For several years the pathways involved in the production of exhaled NO were studied by *in vitro* assays, but the introduction of monoclonal antibodies against cytokines or their receptors allowed us to observe how these directly influence the production of FeNO in humans.

New biological therapies for asthma treatment have helped to elucidate mechanisms that regulate the production of FeNO. For example, in asthmatic patients treated with an IL-4 receptor inhibitor (dupilumab), or an IL-13 inhibitor (lebrikizumab), it is observed a very significant decrease in FeNO levels [34, 49–51], while in asthmatic patients treated with IL-5 inhibitors (mepolizumab), the FeNO levels are not modified [52]. These studies confirmed the experimental evidence that IL-4 and IL-13 are the main cytokines involved in the activation of iNOS and the production of exhaled NO and confirmed that IL-5 is not related with iNOS induction.

While both IL-4/IL-13 and IL-5 are key cytokines of type 2 inflammation, they induce distinct pathways where IL-5 primarily activates STAT-3, while IL-4/IL-13 activates STAT-6. IL-5 induces eosinophilia, but does not contribute to airway NO levels [23, 32]. These three cytokines are expressed together from a common locus of chromosome 5q31 and therefore increased eosinophils in sputum, and high concentrations of FeNO could be often seem together. By reducing eosinophils with antibodies directed to IL-5 or its receptor, there are other cells that still produce IL-4 and IL-13 (e.g., Th2 lymphocytes, mast cells, basophils, and type 2 innate lymphoid cells) that might perpetuate type 2 inflammation and NO production by the bronchial epithelium (Figure 6). In fact, when the IL-4 receptor is blocked in asthmatic patients with a monoclonal antibody, there is a remarkable decrease in FeNO levels in asthmatic patients with elevated eosinophils as well as in patients with low or normal eosinophil counts at the beginning of the study [49]. Treatment with an anti-IgE antibody (omalizumab) also decreases FeNO levels [8, 53, 54] suggesting that activation of IL-4 and IL-13-mediated pathways is crucial in FeNO production.

### 4.1. Applications of FeNO Measurement in Asthma

Several studies have reported that FeNO has a 85% sensitivity and 90% specificity to diagnose asthma, in combination with the clinical history, particularly in patients without steroid treatment and nonsmokers [55–57]. FeNO is also especially useful in patients who are in the early stages of the disease where spirometry changes in reversibility are not yet detected. Schneider et al. analyzed 26 studies with 4,518 patients and concluded that a FeNO <20 ppb has a negative predictive value of 0.86 (95% CI: 0.66-0.95) to exclude the diagnosis of asthma [58]. Recently the GINA guideline suggested that a FeNO above 20 ppb is suggestive of type 2 inflammation which helps to define the endotype as “high type 2 asthma” and with concurrent elevated IgE and allergen sensitization as “allergic asthma” [59, 60]. FeNO measurement is also useful for asthma monitoring and control being levels >30 ppb significantly associated with uncontrolled asthma (*P* = 0.0001) [61, 62].

Another application of FeNO measurement is the prediction of exacerbations in asthmatic patients [62]. This is due to the sensitivity of this biomarker to reflect changes in airway inflammatory conditions and to do so early. In fact, in asthmatic patients who have stopped their steroid treatment, there was a high probability of exacerbation (80–90%) in those with a 10 ppb increase in their FeNO levels on follow-up measurements [63]. Another study found that the majority of asthmatics who experienced exacerbations (76%) had FeNO levels above 28 ppb at baseline [64]. Follow-up with serial FeNO measurements allows early identification of patients without adequate adherence [65]. Smith et al. evaluated the usefulness of FeNO measurements in guiding the therapeutic management of asthma by adjusting corticosteroid doses according to FeNO concentrations [66]. They found that the group of patients monitored with FeNO experienced a 46% reduction in the number of exacerbations and had a statistically significant reduction in the use of inhaled corticosteroids over 12 months [66].

A systematic review of six studies conducted by Essat et al. revealed that asthma treatment in adult patients guided by FeNO levels showed a statistically significant reduction in the number of exacerbations [67]. Most studies to date support the use of FeNO as a biomarker that help to achieve a more effective asthma treatment by minimizing exacerbations and optimizing corticosteroid use [2]. The most recent ATS guidelines of FeNO implementation suggest assessing baseline FeNO levels (baseline determination or first measurement) in comparison to follow-up measurements [68]. An increase or decrease in FeNO greater than 20% of baseline posttreatment is considered clinically significant when baseline levels are greater than 50 ppb. In the case of patients with baseline levels <50 ppb, a difference greater than 10 ppb posttreatment is considered significant [68, 69]. FeNO levels can also be used as biomarker to select the suitability of certain biologic drugs in the treatment of asthma, especially to identify those with type 2 inflammation and allergic asthma [70, 71]. However, it should be interpreted in combination with other type 2 biomarkers such as eosinophil counts, total and specific IgE levels, and the presence of comorbidities and other aspects of the medical history.

### 4.2. Considerations to Consider in the Measurement and Interpretation of FeNO

Although there are differences in cutoff points between some clinical guidelines, FeNO values <25 ppb (or<20 ppb for children) are currently considered to be low or normal, while values >50 ppb (or>35 ppb for children) are highly indicative of type 2 inflammation [72]. Values ranging from 25 to 50 ppb (or 20–35 ppb for children) are considered high but should be interpreted within the clinical context and history of each patient [68]. In recent years, FeNO detection systems have evolved to be practical, robust, portable, and easy to use, so that it is accessible to outpatient clinical practice. However, certain precautions should be taken before measurement as there are several factors that can alter FeNO concentrations. One of the most important is to verify that the patient has not had respiratory infections of viral origin in at least the last three or four weeks before the test. It is also important to know the date of the last exacerbation, since asthma attacks can increase FeNO values well above 100 ppb even when the patient manages levels below that value between crises, so it is suggested to take the measurements at least four weeks after the last exacerbation. This aspect can be controlled with a good medical history and with the evaluation of repeated FeNO measurements in different weeks. Some comorbidities such as allergic rhinitis, aspirin-exacerbated asthma, or nasal polyposis can also increase FeNO values and should be investigated in the anamnesis.

Steroid doses or the “step” of the patient should be also considered as many patients have a result of FeNO levels <25 ppb or<50 ppb but are receiving high doses of inhaled steroids or taking oral steroids. Glucocorticoids decrease FeNO levels even if the patient has a constitutively type 2 inflammation endotype. This implies that of the universe of patients with “high type 2 asthma,” there are those with high FeNO due to insufficient treatment, lack of adherence, or a severe phenotype where type 2 inflammation is not controlled. But there is also a proportion of patients with “high type 2 asthma,” where FeNO can result within normal levels by the effect of corticosteroids. Some authors suggest discontinuing inhaled steroids for at least two weeks before FeNO measurement and taking into account that the fading effect of the steroid on FeNO values ranges from 8 days for fluticasone propionate to 21 days for fluticasone furoate [73].

In addition, age should be considered, since in children, FeNO levels increase to 12 years and then reach levels that are like those in adults [74]. Among the technical indications, patients should be advised not to consume alcohol or tobacco one day before the test [68]. The use of nutritional supplements containing L-arginine or medications containing phosphodiesterase E5 inhibitors should also be investigated as they may increase FeNO levels. Before the test, certain nitrate-rich foods such as spinach or green leafy vegetables should be avoided, since nitrate is reduced to nitrite by bacteria in the oral flora, and by becoming NO by enzymatic and nonenzymatic routes (independent of NOS) could increase FeNO measurements. In contrast, factors that decrease FeNO levels include both short-term and long-term smoking [23].

Although some studies support the use of FeNO in tropical regions [75, 76], more research is still required in patients in those environments to evaluate the role of perennial allergenic exposure and nematode active infections in FeNO measurements [77]. In conclusion, FeNO is a very useful tool in clinical practice that helps to better define the phenotype of asthmatic patients and to monitor the success of treatment and the adherence of the patient, and from the molecular perspective, it is a good indicative of the overexpression of IL-4 and IL-13. Its measurement helps to define better therapeutic approaches within the framework of a more personalized medicine and saves resources by allowing early identification for poorly controlled patients and at risk of exacerbations.

## 5. Conclusions

- Nitric oxide is produced in large quantities by airway bronchial epithelial cells upon upregulation of iNOS. Increased NO is proinflammatory and induces bronchial hyperreactivity and mucus hypersecretion and increases vascular permeability. NO can be measured in the exhaled air as FeNO
- IFN-*γ* induce a physiologic production of NO in the airways, but increased levels of IL-4 and IL13 activate the JAK/STAT-6 pathway altering the intracellular mechanisms that regulate iNOS expression, thus leading to increased FeNO
- FeNO is a robust biomarker of airway inflammation that indicates type 2 inflammation and together with medical history and pulmonary function tests improves asthma diagnosis, helps to identify asthma phenotypes, aids to follow-up treatment response, and is key in choosing personalized treatments

## Figures and Tables

**Figure 1:** Schematic representation of the enzymatic production of nitric oxide (NO) by nitric oxide synthases (NOS) indicating substrate and cofactors.

**Figure 2:** Functions of NO in the airway depending on its concentration from physiological conditions to pathological effects. iNOS: inducible nitric oxide synthase. iNANC: noncholinergic inhibitory noncholinergic.

**Figure 3:** Schematic representation of the homeostatic mechanism of iNOS expression in bronchial epithelial cells under physiological conditions via INF*γ* receptor and the STAT-1 pathway. Once INF*γ* binds its receptor, STAT-1 is phosphorylated and translocated to the nucleus inducing the expression of interferon response factor 1 (*IRF1*) which binds to its response element in the promoter of the *NOS2* gene that encodes for iNOS. Together with the STAT-1 binding elements, they maintain iNOS expression in low concentrations for the physiological production of NO in exhaled air. iNOS promoter also has binding sites for NF*κ*B and AP-1 which increase its expression in response to microbial or environmental signals detected by pattern receptors.

**Figure 4:** Airway diseases that occur with high and low FeNO levels. ppb: parts per billion. AERD: aspirin-exacerbated respiratory disease.

**Figure 5:** Schematic representation of excessive activation of the IL-4/IL-13 receptor and potentiation of STAT-6 signals (red lines) that alter the balance of STAT-1-mediated signals and lead to overexpression of iNOS in patients with type 2 inflammation.

**Figure 6:** Effects of cytokines characteristic of type 2 inflammation on the production of FeNO and other markers of the high T2 asthma phenotype.

## References

[1] Custovic A., Siddiqui S., Saglani S. (2022). Considering biomarkers in asthma disease severity. *The Journal of Allergy and Clinical Immunology*.

[2] Mogensen I., James A., Malinovschi A. (2020). Systemic and breath biomarkers for asthma: an update. *Current Opinion in Allergy and Clinical Immunology*.

[3] American Thoracic S., European Respiratory S. (2005). ATS/ERS recommendations for standardized procedures for the online and offline measurement of exhaled lower respiratory nitric oxide and nasal nitric oxide, 2005. *American Journal of Respiratory and Critical Care Medicine*.

[4] Medrek S. K., Parulekar A. D., Hanania N. A. (2017). Predictive biomarkers for asthma therapy. *Current Allergy and Asthma Reports*.

[5] Sabatelli L., Seppala U., Sastre J., Crater G. (2017). cost-effectiveness and budget impact of routine use of fractional exhaled nitric oxide monitoring for the management of adult asthma patients in Spain. *Journal of Investigational Allergology & Clinical Immunology*.

[6] Beerthuizen T., Voorend-van Bergen S., van den Hout W. B. (2016). Cost-effectiveness of FENO-based and web-based monitoring in paediatric asthma management: a randomised controlled trial. *Thorax*.

[7] Arnold R. J., Massanari M., Lee T. A., Brooks E. (2018). A review of the utility and cost effectiveness of monitoring fractional exhaled nitric oxide (FeNO) in asthma management. *Managed Care*.

[8] Brooks E. A., Massanari M., Hanania N. A., Weiner D. J. (2019). Cost-effectiveness of fractional exhaled nitric oxide (FeNO) measurement in predicting response to omalizumab in asthma. *ClinicoEconomics and Outcomes Research*.

[9] Di Cicco M., Peroni D. G., Ragazzo V., Comberiati P. (2021). Application of exhaled nitric oxide (FeNO) in pediatric asthma. *Current Opinion in Allergy and Clinical Immunology*.

[10] Matsunaga K., Kuwahira I., Hanaoka M. (2021). An official JRS statement: the principles of fractional exhaled nitric oxide (FeNO) measurement and interpretation of the results in clinical practice. *Respiratory Investigation*.

[11] Alahmadi F., Peel A., Keevil B., Niven R., Fowler S. J. (2021). Assessment of adherence to corticosteroids in asthma by drug monitoring or fractional exhaled nitric oxide: a literature review. *Clinical and Experimental Allergy*.

[12] Butler C. A., Heaney L. G. (2021). Fractional exhaled nitric oxide and asthma treatment adherence. *Current Opinion in Allergy and Clinical Immunology*.

[13] Ulrik C. S., Lange P., Hilberg O. (2021). Fractional exhaled nitric oxide as a determinant for the clinical course of asthma: a systematic review. *European Clinical Respiratory Journal*.

[14] Hamada K., Oishi K., Chikumoto A. (2021). Impact of sinus surgery on type 2 airway and systemic inflammation in asthma. *The Journal of Asthma*.

[15] Li Y. H., Yu C. J., Qian X. Y., Song P. P., Gao X. (2021). The correlation between FeNO and nNO in allergic rhinitis and bronchial asthma. *Medicine*.

[16] Antosova M., Bencova A., Mokra D., Plevkova J., Pepucha L., Buday T. (2020). Exhaled and nasal nitric oxide–impact for allergic rhinitis. *Physiological Research*.

[17] Pijnenburg M. W. (2019). The role of FeNO in predicting asthma. *Frontiers in Pediatrics*.

[18] Pijnenburg M. W., De Jongste J. C. (2008). Exhaled nitric oxide in childhood asthma: a review. *Clinical and Experimental Allergy*.

[19] Lu M., Wu B., Che D., Qiao R., Gu H. (2015). FeNO and asthma treatment in children: a systematic review and meta-analysis. *Medicine*.

[20] Tischer C., Karvonen A. M., Kirjavainen P. V. (2021). Early age exposure to moisture and mould is related to FeNO at the age of 6 years. *Pediatric Allergy and Immunology*.

[21] Olivieri M., Marchetti P., Murgia N. (2022). Natural pollen exposure increases in a dose-dependent way fraction of exhaled nitric oxide (FeNO) levels in patients sensitized to one or more pollen species. *Clinical and Translational Allergy*.

[22] Sordillo J. E., Webb T., Kwan D. (2011). Allergen exposure modifies the relation of sensitization to fraction of exhaled nitric oxide levels in children at risk for allergy and asthma. *The Journal of Allergy and Clinical Immunology*.

[23] Hoyte F. C. L., Gross L. M., Katial R. K. (2018). Exhaled nitric oxide: an update. *Immunology and Allergy Clinics of North America*.

[24] Ricciardolo F. L., Sterk P. J., Gaston B., Folkerts G. (2004). Nitric oxide in health and disease of the respiratory system. *Physiological Reviews*.

[25] Forstermann U., Schmidt H. H., Pollock J. S. (1991). Isoforms of nitric oxide synthase Characterization and purification from different cell types. *Biochemical Pharmacology*.

[26] Guo F. H., De Raeve H. R., Rice T. W., Stuehr D. J., Thunnissen F. B., Erzurum S. C. (1995). Continuous nitric oxide synthesis by inducible nitric oxide synthase in normal human airway epithelium in vivo. *Proceedings of the National Academy of Sciences of the United States of America*.

[27] Kobzik L., Bredt D. S., Lowenstein C. J. (1993). Nitric oxide synthase in human and rat lung: immunocytochemical and histochemical localization. *American Journal of Respiratory Cell and Molecular Biology*.

[28] Rosete P. G. L. R., Mancilla B. E., Galindo E. Z. (1999). Óxido Nítrico: Una Molécula Multifuncional. *Revista del Instituto Nacional de Enfermedades Respiratorias*.

[29] Forstermann U., Sessa W. C. (2012). Nitric oxide synthases: regulation and function. *European Heart Journal*.

[30] Yatera K., Mukae H. (2019). Possible pathogenic roles of nitric oxide in asthma. *Respiratory Investigation*.

[31] Uetani K., Thomassen M. J., Erzurum S. C. (2001). Nitric oxide synthase 2 through an autocrine loop via respiratory epithelial cell-derived mediator. *American Journal of Physiology. Lung Cellular and Molecular Physiology*.

[32] Chibana K., Trudeau J. B., Mustovich A. T. (2008). IL-13 induced increases in nitrite levels are primarily driven by increases in inducible nitric oxide synthase as compared with effects on arginases in human primary bronchial epithelial cells. *Clinical and Experimental Allergy*.

[33] Hincapié Díaz M. D. G. A., Lasso Apráez M. D. J. I. (2015). Fracción de óxido nítrico exhalado como biomarcador en asma. *Revista Colombiana de Neumología*.

[34] Alving K., Malinovschi A. (2010). Basic aspects of exhaled nitric oxide. *The European Respiratory Journal*.

[35] Ricciardolo F. L., Sorbello V., Ciprandi G. (2015). FeNO as biomarker for asthma phenotyping and management. *Allergy and Asthma Proceedings*.

[36] Niedbala W., Alves-Filho J. C., Fukada S. Y. (2011). Regulation of type 17 helper T-cell function by nitric oxide during inflammation. *Proceedings of the National Academy of Sciences of the United States of America*.

[37] Wei X. Q., Charles I. G., Smith A. (1995). Altered immune responses in mice lacking inducible nitric oxide synthase. *Nature*.

[38] Negishi T., Kato Y., Ooneda O. (2005). Effects of aryl hydrocarbon receptor signaling on the modulation of TH1/TH2 balance. *Journal of Immunology*.

[39] Niedbala W., Wei X. Q., Piedrafita D., Xu D., Liew F. Y. (1999). Effects of nitric oxide on the induction and differentiation of Th1 cells. *European Journal of Immunology*.

[40] Vig M., Srivastava S., Kandpal U. (2004). Inducible nitric oxide synthase in T cells regulates T cell death and immune memory. *The Journal of Clinical Investigation*.

[41] Yang J., Zhang R., Lu G. (2013). T cell-derived inducible nitric oxide synthase switches off Th17 cell differentiation. *The Journal of Experimental Medicine*.

[42] Niedbala W., Wei X. Q., Campbell C., Thomson D., Komai-Koma M., Liew F. Y. (2002). Nitric oxide preferentially induces type 1 T cell differentiation by selectively up-regulating IL-12 receptor beta 2 expression via cGMP. *Proceedings of the National Academy of Sciences of the United States of America*.

[43] Akata K., Yatera K., Wang K. Y. (2016). Decreased bronchial eosinophilic inflammation and mucus hypersecretion in asthmatic mice lacking all nitric oxide synthase isoforms. *Lung*.

[44] Bentley A. M., Hamid Q., Robinson D. S. (1996). Prednisolone treatment in asthma. Reduction in the numbers of eosinophils, T cells, tryptase-only positive mast cells, and modulation of IL-4, IL-5, and interferon-gamma cytokine gene expression within the bronchial mucosa. *American Journal of Respiratory and Critical Care Medicine*.

[45] Robinson D., Hamid Q., Ying S. (1993). Prednisolone treatment in asthma is associated with modulation of bronchoalveolar lavage cell interleukin-4, interleukin-5, and interferon-gamma cytokine gene expression. *The American Review of Respiratory Disease*.

[46] Guo F. H., Uetani K., Haque S. J. (1997). Interferon gamma and interleukin 4 stimulate prolonged expression of inducible nitric oxide synthase in human airway epithelium through synthesis of soluble mediators. *The Journal of Clinical Investigation*.

[47] Suresh V., Mih J. D., George S. C. (2007). Measurement of IL-13-induced iNOS-derived gas phase nitric oxide in human bronchial epithelial cells. *American Journal of Respiratory Cell and Molecular Biology*.

[48] Modena B. D., Tedrow J. R., Milosevic J. (2014). Gene expression in relation to exhaled nitric oxide identifies novel asthma phenotypes with unique biomolecular pathways. *American Journal of Respiratory and Critical Care Medicine*.

[49] Wenzel S., Castro M., Corren J. (2016). Dupilumab efficacy and safety in adults with uncontrolled persistent asthma despite use of medium-to-high-dose inhaled corticosteroids plus a long-acting *β*_2_ agonist: a randomised double-blind placebo-controlled pivotal phase 2b dose-ranging trial. *Lancet*.

[50] Voraphani N., Gladwin M. T., Contreras A. U. (2014). An airway epithelial iNOS-DUOX2-thyroid peroxidase metabolome drives Th1/Th2 nitrative stress in human severe asthma. *Mucosal Immunology*.

[51] Corren J., Lemanske R. F., Hanania N. A. (2011). Lebrikizumab treatment in adults with asthma. *The New England Journal of Medicine*.

[52] Pavord I. D., Korn S., Howarth P. (2012). Mepolizumab for severe eosinophilic asthma (DREAM): a multicentre, double- blind, placebo-controlled trial. *Lancet*.

[53] Busse W. W. (2019). Biological treatments for severe asthma: a major advance in asthma care. *Allergology International*.

[54] Kurokawa M., Koya T., Takeuchi H. (2020). Association of upper and lower airway eosinophilic inflammation with response to omalizumab in patients with severe asthma. *The Journal of Asthma*.

[55] Guo Z., Wang Y., Xing G., Wang X. (2016). Diagnostic accuracy of fractional exhaled nitric oxide in asthma: a systematic review and meta-analysis of prospective studies. *The Journal of Asthma*.

[56] Dupont L. J., Demedts M. G., Verleden G. M. (2003). Prospective evaluation of the validity of exhaled nitric oxide for the diagnosis of asthma^a^. *Chest*.

[57] Eom S. Y., Lee J. K., Lee Y. J., Hahn Y. S. (2020). Combining spirometry and fractional exhaled nitric oxide improves diagnostic accuracy for childhood asthma. *The Clinical Respiratory Journal*.

[58] Schneider A., Linde K., Reitsma J. B., Steinhauser S., Rucker G. (2017). A novel statistical model for analyzing data of a systematic review generates optimal cutoff values for fractional exhaled nitric oxide for asthma diagnosis. *Journal of Clinical Epidemiology*.

[59] Heffler E., Carpagnano G. E., Favero E. (2020). Fractional exhaled nitric oxide (FENO) in the management of asthma: a position paper of the Italian Respiratory Society (SIP/IRS) and Italian Society of Allergy, Asthma and Clinical Immunology (SIAAIC). *Multidisciplinary Respiratory Medicine*.

[60] Mgaloblishvili N., Gotua M. (2017). Modern approaches to fractional exhaled nitric oxide as a useful biomarker for allergic asthma phenotyping and management. *Georgian Medical News*.

[61] de Abreu F. C., da Silva Junior J. L. R., Rabahi M. F. (2019). The fraction exhaled nitric oxide as a biomarker of asthma control. *Biomarker Insights*.

[62] Menzies-Gow A., Mansur A. H., Brightling C. E. (2020). Clinical utility of fractional exhaled nitric oxide in severe asthma management. *The European Respiratory Journal*.

[63] Jones S. L., Kittelson J., Cowan J. O. (2001). The predictive value of exhaled nitric oxide measurements in assessing changes in asthma control. *American Journal of Respiratory and Critical Care Medicine*.

[64] Gelb A. F., Flynn Taylor C., Shinar C. M., Gutierrez C., Zamel N. (2006). Role of spirometry and exhaled nitric oxide to predict exacerbations in treated asthmatics. *Chest*.

[65] Petsky H. L., Kew K. M., Turner C., Chang A. B., Cochrane Airways Group (2016). Exhaled nitric oxide levels to guide treatment for adults with asthma. *Cochrane Database of Systematic Reviews*.

[66] Smith A. D., Cowan J. O., Brassett K. P., Herbison G. P., Taylor D. R. (2005). Use of exhaled nitric oxide measurements to guide treatment in chronic asthma. *The New England Journal of Medicine*.

[67] Essat M., Harnan S., Gomersall T. (2016). Fractional exhaled nitric oxide for the management of asthma in adults: a systematic review. *The European Respiratory Journal*.

[68] Dweik R. A., Boggs P. B., Erzurum S. C. (2011). An official ATS clinical practice guideline: interpretation of exhaled nitric oxide levels (FENO) for clinical applications. *American Journal of Respiratory and Critical Care Medicine*.

[69] Buchvald F., Eiberg H., Bisgaard H. (2003). Heterogeneity of FeNO response to inhaled steroid in asthmatic children. *Clinical and Experimental Allergy*.

[70] Lee T., Nair P., Corrigan C. J. (2020). Review of monoclonal antibody therapies in asthma and allergic diseases - a new paradigm for precision medicine. *Asian Pacific Journal of Allergy and Immunology*.

[71] Rolla G., Heffler E., Pizzimenti S., Michils A., Malinovschi A. (2020). An emerging role for exhaled nitric oxide in guiding biological treatment in severe asthma. *Current Medicinal Chemistry*.

[72] (2020). GEMA5.0. Guía española para el manejo del asma. *Sociedad Española de Neumología y Cirugía Torácica*.

[73] Lipworth B., Kuo C. R., Chan R. (2020). 2020 updated asthma guidelines: clinical utility of fractional exhaled nitric oxide (Feno) in asthma management. *The Journal of Allergy and Clinical Immunology*.

[74] Buchvald F., Baraldi E., Carraro S. (2005). Measurements of exhaled nitric oxide in healthy subjects age 4 to 17 years. *The Journal of Allergy and Clinical Immunology*.

[75] Cooper P. J., Amoah A. S. (2019). Parasites and allergy: a case of more means less and less means more?. *Parasite Immunology*.

[76] Duenas-Meza E., Torres-Duque C. A., Correa-Vera E. (2018). High prevalence of house dust mite sensitization in children with severe asthma living at high altitude in a tropical country. *Pediatric Pulmonology*.

[77] Pignatti P., Visca D., Loukides S. (2022). A snapshot of exhaled nitric oxide and asthma characteristics: experience from high to low income countries. *Pulmonology*.

